The article "Susceptibility Loci in SLC15A1, UGT1A3, and CWC27 Genes Associated with Bladder Cancer in the Northeast Chinese Population" was retracted in 2023. Reasons: signs of a paper mill; compromised peer review; unreliable results or conclusions.

# Susceptibility Loci in SLC15A1, UGT1A3, and CWC27 Genes Associated with Bladder Cancer in the Northeast Chinese Population

**DOI:** 10.1155/2022/2988159

**Published:** 2022-09-10

**Authors:** Peihong Wu, Yaoxing Guo

**Affiliations:** Department of Pathology, First Affiliated Hospital and College of Basic Medical Sciences of China Medical University, Shenyang 110001, China

## Abstract

Bladder cancer (BCa) is an increasingly severe clinical and public health issue. Therefore, we aim to investigate BCa susceptibility loci in the Chinese population. In this study, 487 BCa patients and 563 controls were recruited from the First Affiliated Hospital of China Medical University from July 2015 to September 2020. A total of ten single-nucleotide polymorphisms (SNPs) in solute carrier family 15 member 1 (SLC15A1), CWC27 spliceosome associated cyclophilin (CWC27), or UDP glucuronosyltransferase family 1 member A3 (UGT1A3) genes were genotyped. The associations between the candidate SNPs and BCa were analyzed using genotype and haplotype analysis. The results demonstrated that Rs4646227 of SLC15A1 has a significant association with BCa. The patients with CG (OR =2.513, *p* < 0.05) and GG (OR =2.859, *p* < 0.05) genotypes had an increasing risk of BCa compared with the CC genotype. For the *CWC27* gene, genotypic frequency analysis revealed that the GT or TT genotype of rs2042329 and the CT or TT genotype of rs1870437 were more frequent in BCa patients than those in the control group, indicating that these genotypes were associated with a higher risk of BCa (all *p* < 0.05). Haplotypes of *SLC15A1*, *UGT1A3*, and *CWC27* genes found that the C-C-C haplotype of *SLC15A1* was associated with a lower risk of BCa while the C-G-C haplotype was associated with a higher risk. For the *UGT1A3* gene, a moderate protective effect was observed with the most frequent T-T-C haplotype, and for the *CWC27* gene, most of the haplotypes showed no association with BCa, except the G-G-C-T haplotype (order of SNPs: rs2042329-rs7735338-rs1870437-rs2278351, OR =0.81, *p* =0.038). In sum, this study indicated that rs2042329 and rs1870437 in the *CWC27* gene and rs4646227 in the *SLC15A1* gene are independent indicators for BCa risk in Chinese people. Further large-scale studies are required to validate these findings. Also, this study provided the theoretical basis for developing new therapeutic drug targeting of BCa.

## 1. Introduction

Bladder cancer (BCa) is the tenth most frequent cancer worldwide with about 573,000 new cases and 213,000 deaths according to the global cancer statistics of 2020 [1]. BCa incidence and mortality rates vary by region and country, and the male incidence is about four times those of women globally [2]. Both environmental factors, such as smoking and occupational exposure [3], and inherited genes or noncoding RNAs are the etiology of BCa [4, 5]. Many genes, including *BIRC5*, *P53*, *BCL2*, *BAX*, *COX2*, *NMP22*, and *MTHFR*, were associated with BCa patients [6].

The article "Susceptibility Loci in SLC15A1, UGT1A3, and CWC27 Genes Associated with Bladder Cancer in the Northeast Chinese Population" was retracted in 2023. Reasons: signs of a paper mill; compromised peer review; unreliable results or conclusions.

Investigating the mechanisms underlying BCa is crucial for improving the screening and diagnosis of BCa [7]. Currently, genome-wide association studies (GWASs) have been done in many populations to identify candidate genes associated to the risk of BCa [8]. A study in Europe demonstrated SNP associations with non–muscle-invasive bladder cancer tumor (size, stage, and grade) and patient characteristics (age and EORTC risk category) at the time of diagnosis [9]. Zhang et al. demonstrate that the minor alleles of rs73862213 and rs2335052 in the GATA2 gene and ZMIZ1 gene were remarkably related with the risk of prostate cancer [8]. Matsuda et al. reported that SNPs in the *SLC14A1*, *APOBEC3A-CBX6*, *PSCA*, and *MYC* genes were associated with the risk of bladder cancer in the Japanese population, and a similar association was demonstrated in Chinese, European, and Asian populations [10]. A Chinese cohort GWAS comprising 3,406 cases of bladder cancer and 4,645 controls identified a new susceptibility locus for BCa in the intron of CWC27 (rs2042329) [11]. SCL15A1, also called PEPT1, was reported to be a highly expressed drug target protein in many different human cancers, including colorectal cancer [12], gastric cancer [13], hepatocarcinoma cells [14], and prostate cancer [15]. SCL15A1 is one of the important molecules during cancer development. Zheng et al. reported that low-frequency variants of UGT1A3 are related with bladder cancer development [16]. Also, UTG1A3 polymorphisms are also associated with patients' drug metabolism [17, 18]. However, replication studies in different populations revealed that only a limited number of loci are definitively associated with the risk of BCa.

To investigate the association between many genes reported in GWASs and the risk of BCa, we performed a replication study in the Chinese population. In this study, 10 loci in *SLC15A1*, *UGT1A3*, and *CWC27* genes were genotyped to determine their association between BCa patients and healthy controls.

## 2. Materials and Methods

### 2.1. Study Population

In this study, 487 BCa patients and 563 controls were recruited from the First Affiliated Hospital of China Medical University from July 2015 to September 2020. The histopathological diagnoses of BCa patients were all evaluated by two pathologists. The healthy controls were individuals who received a physical examination at our hospital. The individuals with a family history of cancer were excluded. After signing the informed consent, a total of 5 mL peripheral blood from all participants was collected for further genotyping. The human ethics committee of the First Affiliated Hospital of China Medical University has approved the whole study.

The article "Susceptibility Loci in SLC15A1, UGT1A3, and CWC27 Genes Associated with Bladder Cancer in the Northeast Chinese Population" was retracted in 2023. Reasons: signs of a paper mill; compromised peer review; unreliable results or conclusions.

### 2.2. Selection of Candidate Genes and SNPs

Three bladder risk-related candidate genes, *SLC15A1*, *UGT1A3*, and *CWC27*, were selected referring to a previous GWAS. Several SNPs were included according to the following criteria: (1) all SNPs were biallelic; (2) SNPs were located in exons or untranslated regions (UTRs) and possibly performing a key function in the development of cancers; (3) the minor allele frequency (MAF) of SNPs in Chinese population is >0.05. In addition, SNPs reported in previous studies were also included. Taken together, a total of ten SNPs in *SLC15A1*, *UGT1A3*, or *CWC27* according to the above criteria were involved in this study (Table 1).

### 2.3. The Genotyping of SNPs

Genomic DNA was isolated from human peripheral blood using TIANamp Genomic DNA Kit (Tiangen Biotech, Beijing, China) according to the manufacturer's standard protocol. Genotyping was performed using the TaqMan SNP genotyping assay on a 7500 Real-Time PCR System (Applied Biosystems, Foster City, CA, USA) according to the manufacturer's instructions. Primers were designed using Primer Express 3.0 software (Applied Biosystems, Foster City, USA). The 20 *μ*L final PCR amplification mix solution contained the following components: 10 *μ*L of master mix (Applied Biosystems), 1 *μ*L of predesigned PCR primers and probes (Applied Biosystems), 50 ng of gDNA, and ddH_2_O. Amplification was carried out as the following conditions: 95°C for 10 sec, followed by 40 cycles of 95°C for 15 sec, and 60°C for 1 min.

### 2.4. Statistical Analysis

Statistical analyses were performed using SPSS software (IBM-SPSS, version 22.0, Chicago, IL, USA). Categorical variables were expressed as percentages and continuous variables were described as means ± SDs. The chi-square statistic test for the control group was used to test the deviation of the Hardy–Weinberg equilibrium. The genotypic association between SNPs and bladder cancer was analyzed using binary logistic regression. Odds ratio (OR) and respective 95% confidence intervals (95% CIs) were calculated to evaluate the effects of different genotypes and alleles. Haplotypes of each gene were analyzed by the SHEsisPlus platform (http://shesisplus.bio-x.cn/SHEsis.html#). The OR results were visualized using GraphPad Prism 6 (https://www.graphpad.com/scientific-software/prism/).

## 3. Results

### 3.1. The Demographic Characteristics of BCa Patients and Controls

The demographic characteristics of 487 BCa patients and 563 controls are summarized in Table 2. The mean age of the BCa and control groups was 64.50 ± 10.56 and 65.05 ± 9.89, respectively. No significant differences in gender (*p* = 0.332) and smoking status (*p* = 0.092) between the two groups were found. Among 487 BCa patients, most (86.2%) were low-grade carcinoma. In addition, 416 (85.4%) BCa patients have non-muscle-invasive tumors, while 71 (14.6%) individuals have invasive tumors.

The article "Susceptibility Loci in SLC15A1, UGT1A3, and CWC27 Genes Associated with Bladder Cancer in the Northeast Chinese Population" was retracted in 2023. Reasons: signs of a paper mill; compromised peer review; unreliable results or conclusions.

### 3.2. The Genotypic Association of Candidate Genes and Bladder Cancer

Analysis of SNP genotype frequency in the control group showed that all candidates' SNPs were in Hardy–Weinberg equilibrium (Table 1). The genotype distribution of SNPs in BCa patients and control groups is provided in Table 3. Furthermore, visualization of the genotype distribution of SNPs is demonstrated in Figure 1. As shown in Table 3 and Figure 1, for three SNPs in the *SLC15A1* gene, only rs4646227 showed a significant association with BCa, whereas no statistical difference was observed for both rs2297322 and rs1289389. The patients with CG (OR =2.513, *p* <0.05) and GG (OR =2.859, *p* <0.05) genotypes had an increasing risk of BCa compared with the CC genotype. Under dominant genotypic model analysis, the OR of CG + GG was 2.545 (*p* <0.05), indicating that rs4646227 were susceptibility loci of BCa. For the *CWC27* gene, both rs2042329 and rs1870437 showed a significant association with BCa. Genotypic frequency analysis revealed that the GT or TT genotype of rs2042329 and the CT or TT genotype of rs1870437 were more frequent in BCa patients than in the control group, indicating that these genotypes were associated with a higher risk of BCa (all *p* <0.05). Similar results were also observed under dominant genotypic model for rs2042329 (OR =1.437, *p* =0.007) and rs1870437 (OR =1.401, *p* =0.011). There is no association between SNPs in *UGT1A3* gene and the risk of BCa.

### 3.3. Haplotype Analysis between Candidate Genes and BCa

Haplotypes of *SLC15A1*, *UGT1A3*, and *CWC27* genes were analyzed using the SHEsisPlus platform in Table 4. Also, the visualization of haplotype distribution of *SLC15A1*, *UGT1A3*, and *CWC27* genes is also demonstrated in Figure 2. As shown in Table 4 and Figure 2, the C-C-C haplotype (order of *SLC15A1* SNPs: rs2297322-rs4646227-rs1289389) of *SLC15A1*, constructed with the C allele of rs4646227, was associated with a lower risk of BCa (OR =0.667, *p* =0.001). In parallel, the C-G-C haplotype, which was constructed with the G allele of rs4646227, was associated with a higher risk (OR =2.231, *p* =0.001). For the *UGT1A3* gene, a moderate protective effect was observed with the most frequent T-T-C haplotype (order of SNPs: rs3821242-rs6431625-rs10929303, OR =0.831, *p* =0.036). For the *CWC27* gene, most of the haplotypes showed no association with BCa, except the G-G-C-T haplotype (order of SNPs: rs2042329-rs7735338-rs1870437-rs2278351, OR =0.81, *p* =0.038).

The article "Susceptibility Loci in SLC15A1, UGT1A3, and CWC27 Genes Associated with Bladder Cancer in the Northeast Chinese Population" was retracted in 2023. Reasons: signs of a paper mill; compromised peer review; unreliable results or conclusions.

Haplotypes with frequency <0.05 are ignored. Order of *SLC15A1* SNPs: rs2297322-rs4646227-rs1289389. Order of *UGT1A3* SNPs: rs3821242-rs6431625-rs10929303. Order of *CWC27* SNPs: rs2042329-rs7735338-rs1870437-rs2278351.

## 4. Discussion

Studies have shown that the occurrence of BCa is associated with the variation of many genes and population heterogeneity [19, 20]. In this study, we investigated several genes previously reported in Chinese and Japanese GWASs to confirm that *SLC15A1* and *CWC27* are genetic factors for BCa.

*SLC15A1* encodes proton-coupled oligopeptide transporter 1 (PEPT1), which is expressed at plasma membranes of epithelial cells in the small intestines and kidneys in mammals [21]. *SLC15A1* is a downstream target gene of the leptin signaling pathway, whose expression is closely associated with obesity and dyslipidemias. In addition, *SLC15A1* was reported to be involved in the diagnosis and therapy of many cancers, including pancreatic cancer [22], bladder cancer [23], gliomas [24], hepatocellular carcinoma [14], renal-cell carcinoma [25], and lung adenocarcinoma [26]. The expression of *SLC15A1* was remarkably lower in metastatic clear-cell renal-cell carcinoma (ccRCC) compared with non-metastatic ccRCC. The expression of *SLC15A1* was downregulated in primary ccRCC compared with that in adjacent kidney normal tissues [25]. *SLC15A1* performs an essential role in the recurrence of lung adenocarcinoma [26]. The three SNPs in the *SLC15A1* gene (rs6491437, rs950905, and rs9557033) showed an increased risk for people with chronic myelogenous leukemia [27]. The rs2297322 of *SLC15A1* was significantly associated with myelosuppression and its subtypes leukopenia and neutropenia [28]. However, the relationship between *SLC15A1* and BCa was still unclear.

In this study, three loci including rs2297322, rs4646227, and rs1289389 in the *SLC15A1* gene were analyzed to examine the association between these SNPs and the risk of BCa in the Chinese population. The CG, GG, and CG + GG genotypes of rs4646227 were correlated with a higher risk of BCa compared with the CC genotype. Interestingly, the haplotype constructed with the G allele (C-G-C) also exhibited a significant association with the occurrence of BCa. In contrast, the C allele (C-C-C) should be potentially protective for BCa. Considering the genotype and haplotype results, rs4646227 should be a potential screen marker for BCa patients.

The article "Susceptibility Loci in SLC15A1, UGT1A3, and CWC27 Genes Associated with Bladder Cancer in the Northeast Chinese Population" was retracted in 2023. Reasons: signs of a paper mill; compromised peer review; unreliable results or conclusions.

*CWC27* is one kind of cyclophilin, which is involved in the binding of proline-containing peptides and participates in protein folding. *CWC27* has an N-terminal PPIase domain containing a proline-binding pocket to bind to proline and a large C-terminal repetitive low complexity region of unknown function [29]. The disruptions of *CWC27* can lead to a spectrum of isolation from syndromic phenotypes, including retinal degeneration, brachydactyly, craniofacial abnormalities, short stature, and neurological defects [30, 31]. Ma et al. [32] reported that CNVs in *CWC27* were related to familial hemangioblastomas. A study showed that SNPs in *CWC27* were associated with the risk of BCa [11]. The T allele of SNP rs2042329, located in intron 1 of *CWC27*, was suggested to be significantly associated with bladder cancer risk in the Chinese population but has no association with Europeans [11]. The effect of rs2042329 on bladder cancer was not associated with age, sex, smoking status, and grades or stages of cancer but was associated with a significantly shorter median recurrence-free time. Also, the rs2042329 T allele was related to significantly higher expression levels of *CWC27* among tumor tissues in low- or high-grade non-muscle-invasive tumors, rather than in the adjacent normal tissues and invasive tumors. A replication study in the UK population [33] also showed that rs2042329 was linked to an increased risk of urinary BCa recurrence.

In this study, four SNPs rs2042329, rs7735388, rs1870437, and rs2278351 in *CWC27* were genotyped in a northeast Chinese population. The results showed that rs2042329 and rs1870437 were significantly associated with a higher risk of BCa, which was consistent with previous reports. The genotype analysis demonstrated that the minor allele of rs2042329 and rs1870437 was significantly associated with the risk of BCa. Due to the few frequencies of the minor allele of the two SNPs, no haplotype was constructed with two T alleles observed. However, the haplotype G-G-C-T, constructed with the G allele of rs2042329 and C allele of rs1870437, showed a protective effect for BCa (OR =0.810, *p* =0.038). These results provide side evidence that *CWC27* is a candidate gene of BCa.

*UGT1A3* encodes a vital protein of the human UDP-glucuronosyltransferase (UGT) superfamily performing a key role in endobiotic and xenobiotic metabolism. Many studies showed that *UGT1A3* was related to many kinds of cancers including pancreatic cancer [34], bladder cancer [16], thyroid cancer [35], stomach cancer [36], colorectal cancer, colon cancer [37], and lung adenocarcinoma [38]. Zheng et al. [16] first revealed that a low-frequency variant rs28898617 in *UGT1A3* was significantly associated with the increased risk of BCa. However, in this study, we failed to replicate the association between SNPs of *UGT1A3* and BCa in the Chinese Northeast population. Neither genotype analysis nor haplotype analysis showed any association with bladder cancer risk.

The article "Susceptibility Loci in SLC15A1, UGT1A3, and CWC27 Genes Associated with Bladder Cancer in the Northeast Chinese Population" was retracted in 2023. Reasons: signs of a paper mill; compromised peer review; unreliable results or conclusions.

In addition, there are some limitations in this study. First, this is a single-center study with a small size of samples. Second, the biological function of the candidate genes was not deeply investigated. The gene–gene or gene–environment interactions were also not determined.

In summary, the association of ten genetic loci in *SLC15A1*, *UGT1A3*, or *CWC27* genes with BCa risk was studied in the Chinese population. The results of our study indicate that rs2042329 and rs1870437 in the *CWC27* gene and rs4646227 in the *SLC15A1* gene are independent indicators for BCa risk in a Chinese population.

Furthermore, large-scale studies are required to validate our findings. Also, cell biological experiments are needed to clarify the tested SNPs that underlie the molecular mechanism and the downstream signaling pathways. Therefore, our study is expected to clarify the molecular mechanism by which this genetic factor contributes to the malignant progression of BCa and provides a theoretical basis for finding new therapeutic targets for BCa.

## Figures and Tables

**Figure 1:** Visualization of the genotype distribution of SNPs in control group and BCa patient group.

**Figure 2:** Visualization of haplotype distribution of *SLC15A1*, *UGT1A3*, and *CWC27* genes in control group and BCa patient group.

**Table 1:** SNP information of *SLC15A1*, *UGT1A3*, or *CWC27.*

Gene	Location	SNPs	Consequence	Allele	MAF in Chinese	HWE *p* in the control group
*SLC15A1*	3q32.2	rs2297322	Exon 5	C/t	0.379	0.173
		rs4646227	Exon 16	C/g	0.104	0.110
		rs1289389	3′ UTR	C/t	0.243	0.413

*UGT1A3*	2q37.1	rs3821242	Exon 1	T/c	0.267	0.823
		rs6431625	Exon 1	T/c	0.121	0.545
		rs10929303	3′ UTR	C/t	0.012	0.086

*CWC27*	5q12.3	rs2042329	Intron 1	G/t	0.141	0.976
		rs7735338	Exon 9	C/g	0.481	0.202
		rs1870437	Intron 10	C/t	0.204	0.280
		rs2278351	Exon 12	T/c	0.476	0.096

**Table 2:** Demographic characteristics of study subjects.

	Cases (*n* =487)	Controls (*n* =563)	*p* values
Age	64.50 ± 10.56	65.05 ± 9.89	0.387
Male (%)	380 (78.0%)	453 (80.5%)	0.332
Smoker (%)	180 (37.0%)	236 (42.1%)	0.092
Tumor grade			
Low	420 (86.2%)	—	—
High	67 (13.8%)	—	—
Clinical stage	232 (47.6%)		
Ta–T1	416 (85.4%)	—	—
T2–T4	71 (14.6%)	—	—

**Table 3:** Genotype distribution of SNPs in BCa patients and control groups.

Gene	SNPs	Genotype	BCa patients	Control groups	OR (95% CI)	*p* value
*SLC15A1*	rs2297322	CC	275	335	—	—
		CT	167	191	1.065 (0.820–1.384)	0.637
		TT	45	37	1.482 (0.932–2.355)	0.095
		CT + TT	212	228	1.133 (0.886–1.448)	0.320
	rs4646227	CC	301	453	—	—
		CG	167	100	2.513 (1.885–3.351)	0.001
		GG	19	10	2.859 (1.311–6.235)	0.006
		CG + GG	186	110	2.545 (1.929–3.358)	0.001
	rs1289389	CC	271	317	—	—
		CT	184	206	1.045 (0.808–1.350)	0.738
		TT	32	40	0.936 (0.572–1.531)	0.792
		CT + TT	216	246	1.027 (0.804–1.311)	0.830

*UGT1A3*	rs3821242	TT	247	304	—	—
		TC	198	218	1.118 (0.866–1.443)	0.392
		CC	42	41	1.261 (0.794–2.001)	0.325
		TC + CC	240	259	1.140 (0.894–1.454)	0.289
	rs6431625	TT	360	435	—	—
		TC	111	118	1.137 (0.847–1.526)	0.394
		CC	16	10	1.933 (0.867–4.313)	0.102
		TC + CC	127	128	1.199 (0.904–1.590)	0.208
	rs10929303	CC	308	367	—	—
		CT	142	167	1.013 (0.773–1.327)	0.924
		TT	37	29	1.520 (0.914–2.530)	0.105
		CT + TT	179	196	1.088 (0.845–1.401)	0.512

*CWC27*	rs2042329	GG	323	416	—	—
		GT	142	136	1.345 (1.020–1.773)	0.035
		TT	22	11	2.576 (1.231–5.389)	0.009
		GT + TT	164	147	1.437 (1.101–1.874)	0.007
	rs7735338	CC	151	161	—	—
		CG	238	294	0.863 (0.652–1.142)	0.303
		GG	98	108	0.968 (0.680–1.376)	0.854
		CG + GG	336	402	0.891 (0.684–1.162)	0.394
	rs1870437	CC	310	400	—	—
		CT	148	145	1.317 (1.003–1.730)	0.048
		TT	29	18	2.079 (1.133–3.813)	0.016
		CT + TT	177	163	1.401 (1.081–1.816)	0.011
	rs2278351	TT	115	139	—	—
		TC	259	301	1.040 (0.772–1.401)	0.796
		CC	113	123	1.110 (0.778–1.584)	0.563
		TC + CC	372	424	1.060 (0.799–1.408)	0.685

The article "Susceptibility Loci in SLC15A1, UGT1A3, and CWC27 Genes Associated with Bladder Cancer in the Northeast Chinese Population" was retracted in 2023. Reasons: signs of a paper mill; compromised peer review; unreliable results or conclusions.

**Table 4:** Haplotype distribution of *SLC15A1*, *UGT1A3*, and *CWC27* genes in the control group and BCa patient group.

Gene	Haplotype	Cases	Controls	OR (95% CI)	*p*
*SLC15A1*	C-C-C	357 (36.6%)	523 (0.464)	0.667 (0.559–0.794)	0.001
	C-C-T	173 (17.7%)	230 (20.4%)	0.841 (0.675–1.047)	0.122
	C-G-C	174 (17.8%)	100 (8.8%)	2.231 (1.715–2.902)	0.001
	T-C-C	179 (18.3)	207 (18.3)	0.999 (0.801–1.247)	0.997

*UGT1A3*	T-T-C	414 (42.5%)	530 (47.0%)	0.831 (0.699–0.988)	0.036
	C-T-C	235 (24.1%)	259 (23.0%)	1.064 (0.869–1.302)	0.544
	T-T-T	156 (16.0)	166 (14.7%)	1.102 (0.869–1.398)	0.419
	T-C-C	98 (10.0%	106 (9.4%)	1.076 (0.806–1.437)	0.617

*CWC27*	G-G-C-T	223 (22.8%)	302 (26.8%)	0.810 (0.664–0.988)	0.038
	G-C-C-C	168 (17.2%)	227 (20.1%)	0.825 (0.661–1.029)	0.088
	G-G-C-C	121 (12.4%)	138 (12.2%)	1.015 (0.782–1.318)	0.907
	G-C-C-T	109 (11.1%)	141 (12.5%)	0.880 (0.674–1.148)	0.347
	T-C-C-C	79 (8.1%)	84 (7.4%)	1.094 (0.795–1.507)	0.578

## Data Availability

The datasets used and analyzed during the current study are available from the corresponding author on reasonable request.
